The article "ANGPTL4 functions as an oncogene through regulation of the ETV5/CDH5/AKT/MMP9 axis to promote angiogenesis in ovarian cancer" was retracted in 2023. Reasons: duplicated images; ethical violations by an author; concerns about the data; concerns about the images.

# ANGPTL4 functions as an oncogene through regulation of the ETV5/CDH5/AKT/MMP9 axis to promote angiogenesis in ovarian cancer

**DOI:** 10.1186/s13048-022-01060-7

**Published:** 2022-12-14

**Authors:** Yinping Liu, Rui Yang, Yan Zhang, Yaping Zhu, Wei Bao

**Affiliations:** 1 Qingpu Branch of Zhongshan Hospital, Fudan University, 1158 Gongyuandong Road, Qingpu District, 201700 Shanghai, P. R. China; 2 Department of Obstetrics and Gynecology, Shanghai General Hospital, Shanghai Jiaotong University School of Medicine, No. 85 Wujin Road, Hongkou, 200080 Shanghai, P. R. China; 3 Department of Obstetrics and Gynecology, Shanghai General Hospital, Shanghai Jiaotong University School of Medicine, No. 85 Wujin Road, Hongkou, 201620 Shanghai, P.R. China

**Keywords:** ANGPTL4, Ovarian cancer, Angiogenesis, CDH5

## Abstract

**Background:**

Angiopoietin-like 4 (ANGPTL4) is highly expressed in a variety of neoplasms and promotes cancer progression. Nevertheless, the mechanism of ANGPTL4 in ovarian cancer (OC) metastasis remains unclear. This study aimeds to explore whether ANGPTL4 regulates OC progression and elucidate the underlying mechanism.

**Methods:**

ANGPTL4 expression in clinical patient tumor samples was determined by immunohistochemistry (IHC) and high-throughput sequencing. ANGPTL4 knockdown (KD) and the addition of exogeneous cANGPTL4 protein were used to investigate its function. An in vivo xenograft tumor experiment was performed by intraperitoneal injection of SKOV3 cells transfected with short hairpin RNAs (shRNAs) targeting ANGPTL4 in nude mice. Western blotting and qRT-PCR were used to detect the levels of ANGPTL4, CDH5, p-AKT, AKT, ETV5, MMP2 and MMP9 in SKOV3 and HO8910 cells transfected with sh-ANGPTL4 or shRNAs targeting ETV5.

**Results:**

Increased levels of ANGPTL4 were associated with poor prognosis and metastasis in OC and induced the angiogenesis and metastasis of OC cells both in vivo and in vitro. This tumorigenic effect was dependent on CDH5, and the expression levels of ANGPTL4 and CDH5 in human OC werepositively correlated. In addition, CDH5 activated p-AKT, and upregulated the expression of MMP2 and MMP9. We also found that the expression of ETV5 was upregulated by ANGPTL4, which could bind the promoter region of CDH5, leading to increased CDH5 expression.

**Conclusion:**

Our data indicated that an increase in the ANGPTL4 level results in increased ETV5 expression in OC, leading to metastasis via activation of the CDH5/AKT/MMP9 signaling pathway.

**Supplementary Information:**

The online version contains supplementary material available at 10.1186/s13048-022-01060-7.

## Introduction

Ovarian cancer (OC) is one the deadliest gynecological tumors [1]. Although surgical and chemotherapy have greatly improved, 80% of patients with advanced high-grade serous OC (HGSOC) will eventually relapse and develop chemotherapy resistant disease, resulting in a 5-year survival rate of 30% [2]. Metastasis is a major cause of recurrence and chemotherapy resistance in OC. The majority of patients with OC are diagnosed at a late stage [2]. However, our knowledge of the key mediators of metastasis process is limited. Therefore, understanding the fundamental mechanisms that drive OC metastasis may lead to the development of effective therapies to reduce morbidity and mortality in patients with OC. Angiogenesis, which is important in tumor metastasis and growth, is a complex and dynamic process involving various molecular regulatory pathways and multiple mechanisms. Antiangiogenic therapy has become an approved therapeutic strategy for several solid tumors. However, for OC patients who receive antiangiogenic therapy, the clinical effect is far from satisfactory [3–6]. There is no doubt that although antiangiogenic therapy is an approved therapeutic strategy for OC, additional potential targets for antiangiogenic therapy need further exploration.

Angiopoietin-like 4 (ANGPTL4) is a secreted protein, that is cleaved into two active peptides; the N-terminal domain is an effective inhibitor of lipoprotein lipase (LPL) activity and regulates lipid composition and energy homeostasis [7]. The C-terminal domain and full-length ANGPTL4 has are involved in vessel permeability, wound healing, and angiogenesis, and promote the progression of a variety of tumors [8–10]. Previous studies have discovered that ANGPTL4 leads to chemotherapy resistance in OC and promotes the progression of OC [11–13]. Previously, ANGPTL4 was reported to promote tumor metastasis and angiogenesis in a variety of tumors [14–16]. Since bevacizumab is not effective in the treatment of OC, it is necessary to further investigate the function of ANGPTL4 in OC and the molecular mechanism by which it promotes angiogenesis. On this basis, our study aimed to systemically verify the biological function of ANGPTL4 in OC using in vivo and in vitro experiments with multiple models, and to explore the underlying molecular mechanisms. Here, we report that ANGPTL4 expression was increased in ovarian tumors and positively correlated with poor prognosis in OC patients. Moreover, downregulating ANGPTL4 dramatically inhibited cancer cell angiogenesis and metastasis both in vitro and in vivo. The tumorigenic effects of ANGPTL4 were elicited via activation of the ETV5/CDH5/p-AKT/MMP9 signaling pathway. These results suggest that ANGPTL4 is a regulator of OC metastasis and angiogenesis.

## Results

### ANGPTL4 is highly expressed in OC and predicts a poor prognosis

To explore the molecular mechanisms of OC metastasis, we performed a high-throughput sequencing analysis of matched metastatic foci and primary foci from OC patients collected from Shanghai General Hospital from April 2017 to December 2018. Differential gene expression was considered to be statistically significant (*P* < 0.05) when the gene copy number was over 2.0-fold and recurred more than three times. Among the differentially expressed genes, ANGPTL4, which has been reported to be highly expressed in a variety of neoplasms and can promote cancer angiogenesis and metastasis, was found to exhibit significantly increased expression in OC metastasis (Fig. 1 A). The protein level of ANGPTL4 was detected by immunohistochemistry (IHC), and we found that ANGPTL4 protein levels were distinctly higher in OC tissue than in normal ovarian tissue (Fig. 1B). Furthermore, we investigated the expression of ANGPTL4 in the normal ovarian cell line Moody and five OC cell lines by real-time PCR and found that the level of ANGPTL4 in the OC cell lines was higher than that in the normal cell line (Fig. 1 C). Consistent with this result, the average levels of ANGPTL4 mRNA in OC tissues were significantly higher than those in normal tissues (Fig. 1D) in TCGA data derived from a total of 580 samples from OCpatients and 8 normal ovarian tissue samples. However, in our paraffin slices and in data from TCGA database, ANGPTL4 expression did not differ significantly between different stages and grades of OC (data not shown). We next sought to determine whether ANGPTL4 expression in human OC is associated with poor survival. We used TCGA database to analyze RNA-seq of 377 patients with OC and divided the patients into the high expression group and the low expression group according to the median expression level in the patients. We found that ANGPTL4 expression was negatively correlated with overall survival (OS, log-rank test *P* = 0.011, HR (95% CI) = 0.71 (0.55–0.93)) (Fig. 1E), the progression-free interval (PFI, log-rank test *p* = 0.026, HR (95% CI) = 0.76 (0.6–0.97)) (Fig. 1 F) and disease-specific survival (DSS, log-rank test *P* = 0.0059, HR (95% CI) = 0.68 (0.51–0.89)) (Fig. 1G). These results suggest that ANGPTL4 expression is upregulated in OC and associated with metastasis and poor prognosis.

**Fig. 1:** ANGPTL4 is highly expressed in OC and OC cell lines. High-throughput sequencing of metastatic and primary sites of OC, with the results shown as a heatmap, Red indicates upregulation and blue indicates downregulation. **B** Representative images of ANGPTL4 immunostaining. ANGPTL4 expression in 18 normal ovarian tissue samples and 97 OC tissue samples was determined by immunostaining. Right panel: the IHC scores for ANGPTL4 in OC and normal ovarian tissues. Analysis of variance (ANOVA) with the post hoc test was carried out, Scale bars, 200 μm. **C** ANGPTL4 mRNA levels in OC cells relative to Moody’s test. Data represent the means ± SD of three independent experiments. **D** ANGPTL4 mRNA expression data in normal ovarian tissue (*n* = 8) and OC tissue (*n* = 580) was retrieved from TCGA. **E**-**G** The overall survival (OS), progression-free interval (PFI) and disease-specific survival (DSS) rates of 377 patients with OC were compared between the low-ANGPTL4 and high-ANGPTL4 groups based on extracted clinical data from TCGA *P < 0.05, **P < 0.01, ***P < 0.001

### ANGPTL4 inhibition attenuates OC metastasis

To verify whether ANGPTL4 can promote the migration and invasion of OC cells, its expression was first silenced in the SKOV3 and HO8910 cell lines using sh-ANGPTL4 expression lentivirus. To explore the role of ANGPTL4 in the metastatic potential of OC in vitro, we first evaluated whether ANGPTL4 affects cell the invasion and migration of OC cells. The results of monolayer wound healing assays (Fig. 2 A) and Transwell chamber migration assays (Fig. 2B) indicated that the migration capacity of ANGPTL4 knockdown (KD) SKOV3 and HO8910 cells was significantly decreased compared with that of the control cells. We further observed a significant decrease in the invasive capacity of ANGPTL4 KD SKOV3 and HO8910 cells compared with the controls, according to the results of Transwell chamber assays (Fig. 2 C). To further confirm the role of ANGPTL4 in promoting metastasis in OC, we conducted xenograft tumor experiments in nude mice. We designed short hairpin RNAs to stably silence ANGPTL4 expression in SKOV3 cells. The extent of the peritoneal metastasis of OC cells was examined by killing nude mice 4 weeks post intraperitoneal injection. ANGPTL4 KD significantly inhibited peritoneal metastasis in mice (Fig. 2D-G). Collectively, the above data showed that ANGPTL4 KD greatly attenuated the metastatic capacity of OC cells.

**Fig. 2:** ANGPTL4 inhibition attenuated OC metastasis. **A** Representative image showing cell migration in the monolayer wound healing assay. Images were obtained at 0 and 24 h after standard wounding. Scale bars, 100 μm. **B** Cell migration assays were performed using 24-well Transwell plates at 24 h after plating. Scale bars, 400 μm. **C** Cell invasion assays were performed using 24-well Transwell plates coated with Matrigel at 24 h after plating. The data are from at least three independent experiments and are shown as the means ± SD. One-way ANOVA. **D** Representative pictures of peritoneal metastasis in a xenograft tumor model generated by the intraperitoneal injection of LV-shCon SKOV3 cells and LV-shANGPTL4 SKOV3 cells (*n* = 8 in each group). **E** Box plot of the weight of metastatic tumor nodules in the abdominal cavities of the groups injected with the LV-shCon SKOV3 cell and LV-shANGPTL4 SKOV3 cell lines. **F** The quantification bar graph shows all implanted nodule volumes in the abdominal cavity of nude mice. **E** Gross morphology of tumor sizes. Scale bars, 100 μm. *P < 0.05; **P < 0.01; ***P < 0.001; NS indicates not significant

### Exogeneous cANGPTL4 protein promotes OC cell progression

The above results suggest that the downregulation of ANGPTL4 expression could inhibit the progression of OC. Consistent with previous studies, ANGPTL4 may play a role in tumorigenesis [17, 18]. We further investigated whether exogeneous cANGPTL4 could facilitate OC metastasis in vitro. We investigated its effect on the migration and invasion of OC cells. In migration assays, OC cells were exposed to the cANGPTL4 protein (250 ng/ml) for 24 h, and the results showed that exogeneous cANGPTL4 significantly increased the migration of both HO8910 and SKOV3 cells (Fig. 3 A-B). In invasion assays, after exposure to exogeneous cANGPTL4 protein (250 ng/ml) for 24 h, the invasive ability of both the HO8910 and SKOV3 cell lines was significantly increased(Fig. 3 C). These results suggest that exogenous cANGPTL4 can promote the functions of OC cells.

**Fig. 3:** Promotion of OC cell progression by incubation with exogeneous cANGPTL4 protein. **A** Treatment with 250 ng/ml rhANGPTL4 increased SKOV3 and HO8910 cell migration compared with that in the PBS group, as shown by Transwell assays. Scale bars, 100 μm. **B** Treatment with 250 ng/ml rhANGPTL4 increased SKOV3 and HO8910 cell migration compared with that in the PBS group, as shown by wound healing assays. Scale bars, 400 μm. **C** Treatment with 250 ng/ml rhANGPTL4 increased SKOV3 and HO8910 cell invasion compared with that in the PBS group, as shown by Transwell assays. Scale bars, 100 μm

### ANGPTL4 promotes OC angiogenesis in vitro

Several studies have shown that ANGPTL4 can promote tumor angiogenesis [19–21]. Considering the importance of angiogenesis in tumor growth and metastasis, the role of ANGPTL4 in OC angiogenesis was further investigated in this study. Thus, we first validated how ANGPTL4 affects angiogenesis by monitoring the tube formation, proliferation, migration, and adhesion abilities of human umbilical vein endothelial cells (HUVECs), which have been widely used as an in vitro model in numerous studies of angiogenesis [22]. First, we used ELISA to detect the expression level of ANGPTL4 in conditioned medium, and the results showed that after ANGPTL4 was knocked out, the expression level of ANGPTL4 in conditioned medium also decreased (Supplementary Fig. 1 A). We investigated whether ANGPTL4 could promote the HUVEC tube formation ability, which involves all steps of angiogenesis. The results showed that conditioned medium (CM) derived from control groups significantly promoted the tube formation ability compared with CM derived from LV-shANGPTL4 groups. At the same time, compared with PBS, treatment with exogeneous cANGPTL4 could enhance the tube formation ability of HUVECs (Fig. 4 A). The migration and proliferation of HUVECs are key steps of angiogenesis [23]. As shown in Fig. 4B, CM derived from LV-Con groups promoted HUVEC proliferation compared with LV-shANGPTL4 groups. In addition, the CM of LV-shANGPTL4 groups could significantly inhibit the migration ability of HUVECs (Fig. 4 C-D). Moreover, treatment with CM derived from LV-Con groups enhanced the adhesion ability of HUVECs (Fig. 4E). At the same time, PBS and recombinant ANGPTL4 were added into the conditioned medium collected by SKOV3 LV-shANGPTL4, respectively, and the results showed that recombinant ANGPTL4 could rescued the tube formation and migration function of HUVEC and protected against ANGPTL4 knockdown-mediated inhibition (Supplementary Fig. 1B-C). These data suggest that ANGPTL4 induces angiogenesis.

**Fig. 4:** ANGPTL4 promotes OC angiogenesis in vitro. **A** LV-shANGPTL4 cell-derived CM inhibited HUVEC tube formation compared with that in the LV-Con groups, and 250 ng/ml rhANGPTL4 treatment increased HUVEC tube formation compared with that in the PBS group, as shown by tube formation assays. Scale bars, 100 μm. **B** LV-shANGPTL4-cell-derived CM decreased the proliferation of HUVECs compared to that in the LV-shCon groups, as characterized by EdU assays. Representative images are shown. Scale bars, 100 μm. **C**-**D** LV-shANGPTL4 cell-derived CM decreased the migration of HUVECs, as shown using the Transwell assay. Representative images are shown Scale bars, 400 μm. **E** Compared to LV-shANGPTL4 CM, CM collected from cells in the LV-shCon group increased HUVEC adhesion. Representative images of attached cells are shown. Scale bars, 100 μm

### ANGPTL4 promotes ovarian cancer angiogenesis in vivo

Next, to explore the role of ANGPTL4 in the angiogenesis of OC in vivo, we chose similarly sized tumor nodules by measuring the microvessel density (MVD) using IHC for CD31. Compared with that in the control group, the number of CD31-positive microvessels in the LV-shANGPTL4 group was significantly reduced (Fig. 5 A). We also detected the correlation between ANGPTL4 levels and MVD in 97 OC patient tissues by IHC staining, and found that the ANGPTL4 level was positively correlated with MVD (Fig. 5B). Examining TCGA OC expression data, we found that the expression of ANGPTL4 was positively correlated with that of CD31 (Fig. 5 C), and we also found that ANGPTL4 expression was positively correlated with that of VEGFA (Fig. 5D). These results suggest that ANGPTL4 is positively correlated with angiogenesis in human OC in vivo and that the expression of ANGPTL4 is independent of VEGFA and cooperatively promotes angiogenesis in OC (Supplementary Fig. 3 A). Consistent with our results, previous studies have also found that both VEGFA and ANGPTL4 are required for angiogenesis [24]. Together, these data suggest that ANGPTL4 stimulates angiogenic activity in OC.

**Fig. 5:** ANGPTL4 promotes OC angiogenesis in vivo. **A** IHC staining of CD31 from the tumors used in Fig. 2D. Representative images from the indicated mice (at least 3 fields per sample and 8 samples per group were quantified). Scale bars, 200 μm. **B** Representative immunohistochemical staining of ANGPTL4 and MVD from 97 paraffin-embedded OC tissues. Scale bars, 200 μm. **C** Correlation of the mRNA expression levels of ANGPTL4 and CD31 from TCGA OC datasets. **D** Correlation of the mRNA expression levels of ANGPTL4 and VEGFA in TCGA OC datasets

### ANGPTL4 promotes OC progression via CDH5

To investigate novel signaling pathways downstream of ANGPTL4 in OC, we subjected all significantly upregulated and downregulated genes (data used in Fig. 1 A) to ingenuity pathway analysis (IPA), and the results suggested that ANGPTL4 interacts with CDH5, further activating AKT and upregulating MMP9 expression (Fig. 6 A). Furthermore, to validate this hypothesis, the mRNA and protein levels of CDH5, AKT, pAKT, MMP9 and MMP2 were detected by RT-qPCR and Western blotting, respectively. The results showed that CDH5 protein and mRNA expression levels in the control group were increased compared with those in the LV-shANGPTL4 group (Fig. 6B-C). CDH5, also known as vascular endothelial cadherin (VE-cadherin), is the major cadherin in endothelial cells, but it is not expressed in the normal epithelium. Many recent studies have demonstrated that CDH5 is highly expressed in tumors and can promote tumor progression. To detect the expression levels of CDH5 in OC and the correlation between ANGPTL4 and CDH5 levels, we used IHC to assess 97 OC samples and found a positive correlation between ANGPTL4 and CDH5 levels (*r* = 0.1215, *P* = 0.0005 Fig. 6D). To evaluate whether the ANGPTL4 promotes SKOV3 cell migration and invasion via CDH5, we stably overexpressed CDH5 in SKOV3 shANGPTL4 cells (Fig. 6E) and performed Transwell assays to evaluate the function of CDH5 in the cells. We found that CDH5 overexpression rescued migration and invasion function and protected against ANGPTL4 KD-mediated inhibition (Fig. 6 F). Consistently, stable KD of ANGPTL4 inhibited pAKT, MMP9 and MMP2 expression at both the protein and mRNA levels in the HO8910 and SKOV3 cell lines, but MMP2 mRNA levels in the SKOV3 cell lines were not significantly different upon ANGPTL4 KD (Fig. 6G-I). These results suggest that ANGPTL4 promotes the migration and invasion of OC cells through the upregulation of CDH5.

**Fig. 6:** ANGPTL4 promotes OC progression via CDH5. **A** Top network identified by IPA. Gene signatures of metastatic sites and primary sites of OC. **B** CDH5 protein levels in HO8910 and SKOV3 cells with stable ANGPTL4 KD were analyzed by Western blotting. **C** CDH5 mRNA levels in HO8910 and SKOV3 cells with stable ANGPTL4 KD were analyzed by RT–qPCR. **D** Representative immunohistochemical staining of ANGPTL4 and CDH5 in 97 OC tissues. Correlation of the expression levels of ANGPTL4 and CDH5 in 97 OC tissues. (*r* = 0.1643, *p* < 0.0001), Scale bars, 200 μm. **E** The effect of gene vector delivery on CDH5 mRNA levels was assessed by RT-PCR; the bar graph shows the mean fold change over data from the control (*n* = 3). **F** Cell migration and invasion assays were performed using 24-well Transwell plates at 24 h after plating. These data are from at least three independent experiments and are shown as the means ± SD. One-way ANOVA. Scale bars, 400 μm. **G** The indicated cells stably transfected with control or ANGPTL4 shRNA were used to analyze protein levels by Western blotting. H-I. The indicated cells stably transfected with control or ANGPTL4 shRNA were used to analyze the mRNA levels of the indicated molecules by qRT-PCR

### ANGPTL4-induced upregulation of CDH5 expression is modulated by ETV5

It has been reported that cANGPTL4 directly interacts with VE-cadherin on endothelial cells to induce vascular leakiness, leading to tumor metastasis [17]. To determine whether ANGPTL4 directly binds CDH5 in OC cells to initiate downstream signaling pathways, we used coimmunoprecipitation (CoIP) experiments, and the results suggested that the two are not directly related (Fig. 7 A). To further understand how ANGPTL4 affects CDH5 expression in OC, global transcriptomics analysis was carried out in SKOV3 and H08910 cells in which ANGPTL4 was stably knocked down, and the global transcriptomes were compared with those from cells transfected with control lentivirus. Intriguingly, we found nearly 226 genes in both the SKOV3 and HO8910 control cell lines that were more than 2-fold higher in abundance than those in ANGPTL4 KD cells (Fig. 7B). Among them, Ets variant gene 5(ETV5), a transcription factor in the ETS family, has been found to promote metastatic progression in several types of human cancers [25–27]. Members of this family, including Erg and Ets-1, bind the VE-cadherin promoter and enhance activity [28, 29]. Based on these studies, we hypothesized that ETV5 may affect the transcription of the upstream promoter region of the CDH5 gene, thereby interfering with the expression of downstream genes. Furthermore, to validate this hypothesis, we first detected differences in the ETV5 protein level between the LV-Con and LV-shANGPTL4 groups, and the results showed that the ETV5 protein level was lower in the LV-shANGPTL4 groups (Fig. 7 C), as suggested by analysis with the Jaspar website (http://jaspar.genereg.net/analysis) (Supplementary Fig. 2B ); this result was subsequently confirmed by a chromatin immunoprecipitation (ChIP) assay. These data showed that ETV5 can bind the promoter region (-959-799 bp, -782-569 bp and − 465 − 209 bp) of CDH5 (Fig. 7D). Therefore, ETV5 promotes CDH5 expression through the transcriptional activation of CDH5. We additionally transfected ETV5 siRNA into two OC cell lines (SKOV3 and HO8910), and we found that ETV5 siRNA downregulated the expression of CDH5 (Fig. 7E). On the other hand, we overexpressed ETV5 in the LV-shANGPTL4 SKOV3 cell line and detected expression changes in the target protein. We found that the expression of ANGPTL4 was not significantly affected, while the expression levels of CDH5, p-Akt and MMP9 were increased (Fig. 7 F). Taken together, these results indicate that ANGPTL4 might regulate CDH5 via ETV5.

**Fig. 7:** ANGPTL4 upregulation of CDH5 expression is modulated by ETV5. **A **Results of Co-IP analysis of ANGPTL4 and CDH5 levels detected by Western blotting. **B** A heatmap showing differentially regulated genes in SKOV3 cells and HO8910 cells transfected with control or ANGPTL4 shRNA. The color scheme is shown beside the data. **C** ETV5 protein levels in HO8910 and SKOV3 cells with stable ANGPTL4 KD were analyzed by Western blotting. **D** ChIP-qPCR analysis of ETV5 binding at loci 1, 2, 3, 4, and 5. The means ± SDs of triplicate experiments are shown. *P < 0.05, **P < 0.01, ***P < 0.001. **E** CDH5 protein levels were determined by Western blotting after ETV5 expression was downregulated. **F** The protein levels of ANGPTL4, ETV5, CDH5, p-AKT and MMP9 in LV-shANGPTL4 SKOV3 cells were analyzed by Western blotting

## Discussion

An increasing number of studies have shown that ANGPTL4 plays an important role in the occurrence and development of cancer. At the same time, several studies have reported conflicting roles for ANGPTL4 in cancer. For example, ANGPTL4 was found to be upregulated in tumor tissues and promotes tumor angiogenesis and metastasis [19, 30, 31]. In contrast, another study found that ANGPTL4 expression was significantly lower in HCC tissue than in adjacent normal liver tissue and that ANGPTL4 inhibited tumor angiogenesis and metastasis [32]. H-Y Hsieh et al. revealed that ANGPTL4 has dual roles in the progression of urothelial carcinoma, acting as either an oncogene or tumor suppressor [33]. However, whether ANGPTL4 behaves as an oncogene or a tumor suppressor depends on the cancer tissue type [9]. Several studies have demonstrated that ANGPTL4 is overexpressed in OC and that this overexpression is related to shorter relapse-free survival times in serous OC [13, 34, 35].On this basis, we wanted to further verify the biological function and molecular mechanism of ANGPTL4 in OC. Our initial observations focused on the abnormally high expression of ANGPTL4 in metastatic OC foci compared with primary foci using high-throughput sequencing. Then, we found that ANGPTL4 expression was upregulated in OC tissue compared with normal ovarian tissue and significantly correlated with a poorer prognosis in OC patients (Fig. 1).

Based on the above results, it is reasonable to propose that ANGPTL4 plays an important role in the progression of OC. We found that downregulating ANGPTL4 expression inhibited OC metastasis both in vitro and in vivo (Fig. 2); at the same time, rhANGPTL4 stimulated OC cell metastasis and invasion (Fig. 3). In addition to our research, several other studies have reported that high ANGPTL4 expression could promote the metastasis of breast cancer [10], gastric cancer [36], cutaneous melanoma [37], head and neck squamous cell carcinoma [38], and others. Many studies have revealed that angiogenesis plays a vital role in cancer development and is an essential part of the metastasis of many solid tumors, and the inhibition of angiogenesis has become a recognized therapeutic strategy for many solid tumors, including OC [39–41]. Herein, our study indicated that ANGPTL4 could promote OC angiogenesis both in vitro and in vivo (Figs. 4 and 5). We also found that the expression level of ANGPTL4 was independent of VEGFA expression. (Supplementary Fig. 3 A-B). Bevacizumab is a humanized anti-VEGF monoclonal antibody that was approved by the FDA for the treatment of OC, but the results with this antibody have been disappointing. Here, we identified ANGPTL4, a different angiogenic factor in OC. Previous studies have shown that high ANGPTL4 expression is correlated with a poor response to anti-VEGF therapies [42]. In addition, J. Incio et al. reported elevated ANGPTL4 expression as another mechanism of resistance to anti-VEGF therapies in obese mice [43]. Therefore, targeting ANGPTL4 alone or in combination with anti-VEGF treatment may be a better therapeutic option for OC patients.

ANGPTLs are orphan ligands because they do not bind either the angiogenic receptor tyrosine kinase Tie2 or VEGFR [44]. The biological function of ANGPTL4 has been reported to be predominantly related to cell metastasis and angiogenesis as ANGPTL4 has been shown to target fibronectin, Myc, NFKB, and 14-3-3γ. Wen-Hsuan Yang reported that in OC, the TAZ-ANGPTL4-NOX2 axis regulates chemotherapy resistance [12]. Yuxian Wu and coworkers suggested that the VEGFR2 pY949/VE-cadherin/Src pY416 complex plays a role in regulating vascular integrity [13]. Here we report that CDH5 is responsible for mediating the metastasis and angiogenic function of ANGPTL4, as the restoration of CDH5 levels was found to elicit a rescue effect. CDH5, also known as VE-cadherin, is a cell-surface adherent protein that connects cancer cells with extracellular domains to form tumor blood vessels [45, 46]. In normal tissues and cells, VE-cadherin i expression is restricted to vascular endothelial cells, and VE-cadherin is not expressed in various other normal tissues and cells; however, VE-cadherin is aberrantly overexpressed in various malignant tumors [45, 47, 48] and has been found to promote tumor metastasis. In this study, we observed that CDH5 was expressed in OC epithelial tissues and that CDH5 expression was dysregulated by ANGPTL4 overexpression. However, how ANGPTL4 regulates CDH5 was unknown. Through integrative analyses in this study, we found that ETV5 could directly bind the promoter regions of CDH5, which was upregulated by ANGPTL4 in OC cells. ETV5 belongs to the ETS family, which has been associated with the progression and invasion of tumors and is important for vasculogenesis and angiogenesis [49]. Among the members of this family, Erg and Ets-1 can bind the CDH5 promoter and enhance its activity [28, 29]. Here, we found with ChIP assays that ETV5 upregulates CDH5 expression and that directly binds the CDH5 promoter region. Importantly, both CDH5 and ETV5 have been shown to be associated with poor prognosis in multiple cancer types [25, 50–52]. However, we also found that blocking ANGPTL4 in OC cells inhibited the phosphorylation of AKT, MMP9 and MMP2, which plays an important role in tumor progression and metastasis.

In summary, the results of our study provide in vivo and in vitro evidence to support the pro-oncogenic function of ANGPTL4 in the metastasis of OC and advance our understanding of the mechanism by which ANGPTL4 regulates ovarian tumor metastasis. The major findings of the present study are summarized in a diagram (Supplementary Fig. 3 C). Elevated ANGPTL4 expression in OC increases the expression of CDH5 by upregulating ETV5, which can bind the CDH5 promoter region and activate AKT, followed by the induction of MMP9. Moreover, increased expression of ANGPTL4 can promote angiogenesis in OC. In conclusion, our results revealed the biological function and mechanism of ANGPTL4 in OC, which may be a novel candidate therapeutic target for metastatic OC.

## Materials and methods

### Cell culture and transfection

The human OC cell lines SKOV3, H08910, Hey, A2780 and A2780/DDP (cisplatin-resistant cell line) were cultured in RPMI 1640 (Gibco, Auckland, New Zealand) medium. SKOV3 cells were obtained from the FuHeng Cell Center (Shanghai, China). HO8910 cells were obtained from Procell Life Science & Technology. An immortalized ovarian epithelial cell line (Moody) and HUVECs were conserved in our laboratory and had been purchased from the American Type Culture Collection (ATCC), these cell lines were cultured in DMEM:F12 (1:1, Gibco). All cell lines were cultured according to standard protocols and maintained at 37 °C under 5% CO_2_. Prior to the beginning of the experiment, we have carried out STR certification on the relevant cell lines. ANGPTL4 KD was achieved by transfecting lentiviral (Lv) plasmids expressing shRNAs targeting ANGPTL4 into OC cells. ETV5 short interfering (si)RNA and negative controls were purchased from RiboBio (Guangzhou, China). We obtained shANGPTL4 plasmids and negative controls from OBIO (Shanghai, China). The protocols involving all cell lines received ethical approval from the Human Research Ethics Committee of Shanghai General Hospital affiliated to Shanghai Jiao Tong University.

## Patients and sample collection

The tissue microarray (TMA) included 97 OC tissues and 2 normal ovarian tissues and was purchased from the Shanghai Weiao Biological Company. Eighteen normal ovarian tissue samples were collected from the Department of Gynecology and Obstetrics, Shanghai General Hospital, between 2018 and 2019. Four pairs of metastatic foci and primary foci from OC samples were collected for high-throughput sequencing after surgery at Shanghai General Hospital from April 2017 to December 2018. None of the patients received any preoperative treatment. Samples were cryopreserved in liquid nitrogen. All patients signed informed consent forms. This study was approved by the Institutional Research Ethics Committee of Shanghai General Hospital.

### High-throughput sequencing of mRNAs

Total RNA was isolated using an RNeasy mini kit (Qiagen, Germany). The TruSeq™ RNA Sample Preparation Kit (Illumina, USA) was used to synthesize the paired-end library according to instructions in the sample preparation guide. The library was constructed and sequenced by Sinotech Genomics Co., Ltd. (Shanghai, China). Differential mRNA expression was analyzed by R language packages. Differentially expressed RNAs with a |log2(FC)| value > 1 and a q value < 0.05 were regarded as significantly differentially expressed.

### Lentiviruses and reagents

Lentivirus vectors encoding human shRNAs against ANGPTL4 and an empty vector (LV-shCon) were purchased from OBIO (Shanghai, China). Cells were stably transfected with lentivirus, grown and harvested after puromycin selection for 14 days. Details of the commercial antibodies are shown in Table 1.

**Table 1:** Detailed information of our commercial antibodies

Antibody	Concentration for WB	Concentration for IHC	Company
GAPDH (ab181602)	1: 10,000		Abcam
CD31 (ab182981)		1: 400	Abcam
CDH5(ab33168)	1: 1000	1: 50	Abcam
ANGPTL4(ab196746)	1: 1000	1: 100	Abcam
MMP9 (#13,667)	1:1000		Cell Signaling Technology
AKT(#4685)	1: 1000		Cell Signaling Technology
pAkt(#4060)	1: 2000		Cell Signaling Technology
ETV5 (66657-1-lg)	1:1000		Protein Tech
MMP2(#13,132)	1: 1000		Cell Signaling Technology

### Real-time PCR

Using TRIzol reagent (TaKaRa, Japan), total RNA was isolated according to the manufacturer’s instructions, and qRT-PCR was performed with TB Green Premix Ex Taq (TaKaRa, Japan) on a 7500 real-time PCR system (AB Applied Biosystems, Germany) and was determined by the 2^−ΔΔCt^ method. All primers sequences used are shown in Table 2.

**Table 2:** Primers used for qRT-PCR

Gene name	forward(5’-3’)	reverse(5’-3’)
GAPDH	CGTATTGGGCGCCTGGTCAC	ATGATGACCCTTTTGGCTCC
ANGPTL4	GTCCACCGACCTCCCGTTA	CCTCATGGTCTAGGTGCTTGT
CDH5	TTGGAACCAGATGCACATTGAT	TCTTGCGACTCACGCTTGAC
MMP2	TACAGGATCATTGGCTACACACC	GGTCACATCGCTCCAGACT
MMP9	TGTACCGCTATGGTTACACTCG	GGCAGGGACAGTTGCTTCT
VEGFA	AGGGCAGAATCATCACGAAGT	AGGGTCTCGATTGGATGGCA

### Western blot analysis

Cellular extracts containing the same amount of protein were separated on SDS-polyacrylamide mini-gels and transferred to PVDF membranes (Millipore, Billerica, MA, USA) for 90 min at 300 mA. The membranes were blocked with 5% skim milk at room temperature for 1 h and then incubated with specific primary antibodies at 4 °C overnight. Then, they were washed with TBST buffer3 times (10 min each) and incubated with secondary antibodies (1:5000 dilution; Proteintech, Chicago, 1 L) at room temperature for 1 h. ECL chemiluminescence (Millipore) was used to detect proteins.

### IHC

ANGPTL4, CDH5 and MVD-related protein levels were analyzed by IHC as previously reported [53]. The percentage of positive cells was scored as follows: 1) The staining area score was calculated as follows: 0′, < 5%; 1′, 5–25%; 2′, 26–50%; 3′, > 51–75%; and 4’, > 76%. 2) The staining intensity score was calculated as follows: 0′, no staining; 1′, mild staining; 2′, moderate staining; and 3′, intense staining. 3) Total staining score based on both the staining area and intensity.

### Transwell and wound healing assays

For Transwell migration assays, 1 × 10^5^ cells/100 µl were seeded in the upper chambers of 24-well plates (8 µmol pores, Corning, NY, USA) with serum-free medium. RPMI 1640 medium containing 10% FBS was added to the lower chamber. After 24 h, the cells in the upper part of the chamber were removed, and the cells in the lower part of the chamber were fixed with formaldehyde and stained with crystal violet. In the invasion test, the upper chamber was precoated with Matrigel (BD Biosciences, CA), and cells were seeded in the upper chamber in serum-free medium. Medium containing 10% serum was added to the lower chamber. After 48 h, invaded cells were fixed and stained with crystal violet. The cells were counted under a microscope.

HUVEC migration assay was performed using Falcon™ Cell Culture Inserts (BD353097) according to the manufacturer’s instructions. Then, 200 µl of serum-free medium containing 1 × 10^5^ HUVECs was added to the upper chamber, and 800 µl tumor supernatant was added to the lower chamber and incubated at 37 °C with 5% CO_2_ for 24 h. Cells were incubated with a subsequent tumor procedure as previously described.

The wound healing experiment was performed by plating 1 × 10^5^ cells per well in 6-well plates, a 100 µl pipette tip was used to create 3 wounds devoid of cells, and medium without FBS was added. Images were captured at 0 and 24 h, and wound widths were quantified and compared to baseline values.

### Cell proliferation assay

The proliferative ability of HUVECs after coculture with CM from different cells was determined by an EdU proliferation assay (RiboBio). After pretreatment as described above, HUVECs were incubated in 50 M EdU for 2 h and then fixed, permeabilized, and stained following the manufacturer’s instructions.

### Endothelial tube formation assay

HUVECs at a density of 1 × 10^4^ cells/well in 96-well plates were cultured in 250 ng/ml rhANGPTL4 or tumor supernatants from each cell line for 6 h. The plates were precoated with 100 µl of Matrigel (BD Bioscience) at 37 °C for 1 h. After 6 h of incubation, images of the tubules were acquired and analyzed by Image-Pro Plus software and tubules were quantified by counting the number of tubes in 10 randomly chosen fields of view. Data were obtained from three independent experiments.

### Analysis of human OC data from TCGA

ANGPTL4 expression data in OC were retrieved from TCGA (580 OC patient samples and 8 normal ovarian tissues). Then, the correlation between ANGPTL4 expression and CD31 expression and the correlation between ANGPTL4 expression and VEGFA expression were assessed. Survival curves were determined by the Kaplan-Meier method with the website: http://www.kmplot.com. Progression-free survival (PFI, *n* = 377), disease-specific survival (DSS, *n* = 377) and overall survival (OS, *n* = 377) were analyzed using TCGA data.

### CoIP assay

For CoIP assays, SKOV3 cells were lysed on ice in lysis buffer (20 mM Tris HCl, pH = 8, 137 mM NaCl, 10% glycerol, 1% Nonidet P-40, 2 mM EDTA and protease inhibitor) for 30 min with occasional vortexing, and centrifugation was performed for 12 min to remove cellular debris. After preclearing, 500 µl of protein lysate was immunoprecipitated with anti-CDH5 antibody (Abcam, ab33168) and protein A Sepharose beads. The immunoprecipitates were then probed with anti-ANGTPL4 (Santa Cruz Biotechnology, SC-373,761) and anti-CDH5 (Abcam, ab33168) antibodies. The precipitates were separated by SDS-PAGE and analyzed by immunoblotting.

### ChIP assays

ChIP assays were performed with a ChIP Kit (Millipore) following the manufacturer’s protocol. Protein and DNA were crosslinked in 1% formaldehyde, with glycine used to terminate the crosslinking reaction, after which the crosslinked molecules were extracted with SDS lysis buffer, and sheared by sonication. An ETV5 antibody (Proteintech 66657-1-lg) was used for immunoprecipitation. After purification of the precipitated DNA, PCR was conducted. The primer sequences used for PCR are listed in Table 3.

**Table 3:** The primers used for PCR of CHIP assay

number	Primer name	nucleotide sequences(5’to 3’)
1	CDH5 promoter-1-F	CCCCAAATGTCAGAGGGTCC
2	CDH5 promoter-1-R	GACCCTGAGAAAGAGAGGGC
3	CDH5 promoter-2-F	AGATTCCCAGGATCTGCCCT
4	CDH5 promoter-2-R	GCTGGATCAGAGCCCAGAAG
5	CDH5 promoter-3-F	TCCACGCCCCTCTTTGATTC
6	CDH5 promoter-3-R	GACTCCAGCTCTAAGGTGCC
7	CDH5 promoter-4-F	CCCACAAAGACATCATGGGA
8	CDH5 promoter-4-R	CAGCTCTGGGACTCTGAACC
9	CDH5 promoter-5-F	GAAAACCTGAAGGGGAGGCA
10	CDH5 promoter-5-R	TGTGGGCTGAGGGATGTTTC

### Tumor xenograft mouse model

All animal experiments were carried out in strict accordance with the Guide for the Care and Use of Laboratory Animals and approved by the Department of Laboratory Animal Science, School of Medicine, Shanghai Jiao Tong University. SKOV3-LV-shCon and SKOV3-LV-shANGPTL4 cells (5 × 10^6^ cells/100 µl) were intraperitoneally (i.p.) injected into 5-week-old BALB/c nu/nu female mice (8 mice per group). After 4 weeks, the animals were anesthetized and killed with an excess of 2% pentobarbital sodium (0.5 ml), and death was then confirmed with cervical dislocation. The intraperitoneal tumor nodules were extracted and weighed.

### ELISA

A Human ANGPTL4 ELISA kit (RAB0017, Sigma Aldrich) was used as instructed by the manufacturer quantify the secretion of ANGPTL4 in cell culture medium.

### CM

Control and LV-shANGPTL4 groups of SKOV3 and HO8910 cells were seeded at a density of 1 × 106 in 60-mm Petri dishes and cultured in RPMI 1640 medium for 48 h. The CM was collected and centrifuged at 3000 rpm for 10 min at 4 °C.

### Statistical analysis

All data are presented as the means ± SD. Data from two groups were compared by two-tailed Student’s t-test. GraphPad Prism 6.0 (GraphPad Software, Inc., La Jolla, CA, USA) was used for all statistical analyses. Differences for which the P value was < 0.05 were considered statistically significant.

## Supplementary Information

**Additional file 1:** **Supplementary Figure 1. **A. ELISAshowing the level of extracellular ANGPTL4 proteins in the culture media ofSKOV3 cells and HO8910 cells transfected with control or ANGPTL4 shRNA andincubated for 2 days (Student’s *t*-test; ***p < 0.0001). B. Recombinant ANGPTL4 rescued changes in HUVEC tube formation activity due to treatment with LV-SKOV3-shANGPTL4 CMas shown using the tube formation assay. Representative images are shown. Scale bars, 400 µm.C. Recombinant ANGPTL4 rescued changes in HUVEC migration activity due totreatment with LV-SKOV3-shANGPTL4 CM as shown using the transwell assay.Representative images are shown. Scale bars, 100 µm. **Supplementary Figure 2. **A.Top network identified by IPA. Gene signatures of metastatic sites and primarysites of OC. B. The binding sites of ETV5 to the CDH5 promoter as predicted bythe online Jaspar website (http://jaspar.generge.net/). **Supplementary Figure 3. **The expression level ofANGPTL4 is independent of each other with VEGFA. A. VEGFA mRNA expression level after knock downANGPTL4 in OC cells. Data represent mean±SD of three independent experiments.B. Expression level of ANGPTL4 after adding 250ng/ml bevacizumab in OC cellculture medium. Data represent mean±SD of three independent experiments. C. Anelevated ANGPTL4 in ovarian cancer increases the expression of CDH5 byup-regulating ETV5 which could binding to CDH5 promoter region, would activateAKT followed by induction of MMP9. At the same time, high expression of ANGPTL4can promote angiogenesis of ovarian cancer. 

**Additional file 2. **

**Additional file 3.**

**Additional file 4.**

## Data Availability

All data generated or analyzed during this study are included in this published article [and its supplementary information files].

## Abbreviations

HGSOC: High-grade serous ovarian cancer
ANGPTL4: Angiopoietin-like 4
HUVECs: Human umbilical vein endothelial cells
CDH5: Cadherin 5
ETV5: ETS variant 5
